The article "Meta-Analysis of Low Temperature Plasma Radiofrequency Ablation and CO2 Laser Surgery on Early Glottic Laryngeal Carcinoma" was published in 2022. Journal: Comput Math Methods Med.

# Meta-Analysis of Low Temperature Plasma Radiofrequency Ablation and CO_2_ Laser Surgery on Early Glottic Laryngeal Carcinoma

**DOI:** 10.1155/2022/3417005

**Published:** 2022-07-06

**Authors:** Cheng Wang, Ye Zhao, Changhu Li, Qiang Song, Fuxing Wang

**Affiliations:** ^1^Krirk University, Thailand; ^2^Tianjin Liyuan Medical Technology Co., Ltd., China; ^3^Shandong University of Traditional Chinese Medicine, China

## Abstract

**Objective:**

Meta-analysis is used to analyze the treatment of early glottic laryngeal carcinoma by cryogenic plasma radiofrequency ablation combined with CO_2_ laser surgery.

**Methods:**

Retrieval of PubMed, Embase, Medline, VIP, Wanfang, and CNKI databases using a computer. The retrieval period is from the creation of the database until August 31, 2021. References to the included literature were also searched at the same time. According to the inclusion and exclusion criteria, literatures are screened independently, relevant data were extracted, and meta-analysis was conducted.

**Results:**

Recurrence rates are reported in seven literatures. In interstudy heterogeneity test: *P* = 0.624, *I*^2^ = 0%, fixed effect model analysis shows that there is no significant difference in recurrence rate between low temperature plasma radiofrequency ablation and CO_2_ laser ablation (OR = 0.80, 95% CI (0.35, 1.29), *P* = 0.371). Intraoperative blood loss is reported in 5 literatures, and heterogeneity test of each study is as follows: *P* = 0.03, *I*^2^ = 67%. Low temperature plasma radiofrequency ablation results in more intraoperative blood loss than CO_2_ laser ablation (SMD = −0.71, 95% CI (0.08, 0.82), *P* = 0.01). There are five reports on postoperative pain in two treatments: *P* = 0.04, *I*^2^ = 64%. There is no significant difference in postoperative pain between low temperature plasma radiofrequency ablation and CO_2_ laser ablation (SMD = −0.21, 95% CI (-0.44, 0.10), *P* = 0.134). Operative time is reported in nine articles: *P* < 0.01, *I*^2^ = 95%. The operative time of low temperature plasma radiofrequency ablation is significantly shorter than CO_2_ laser ablation (SMD = −2.38, 95% CI (-3.91, -1.62), *P* < 0.01). There are two reports on postoperative mucosal recovery: *P* = 0.328, *I*^2^ = 2%. Low temperature plasma radiofrequency ablation was significantly better than CO_2_ laser ablation in postoperative mucosal recovery (OR = 5.49, 95% CI (2.36, 10.18), *P* < 0.01).

**Conclusion:**

Low temperature plasma radiofrequency ablation is superior to CO_2_ laser surgery in the treatment of early glottic laryngeal carcinoma in terms of operative time and postoperative mucosal recovery. Low-temperature plasma radiofrequency ablation, on the other hand, results in higher intraoperative blood loss, with no discernible difference in recurrence rate or postoperative pain severity between the two treatments.

The article "Meta-Analysis of Low Temperature Plasma Radiofrequency Ablation and CO2 Laser Surgery on Early Glottic Laryngeal Carcinoma" was published in 2022. Journal: Comput Math Methods Med.

## 1. Introduction

Laryngeal cancer is a common tumor in otorhinolaryngology, accounting for 1% ~5% of all malignant tumors. The total incidence of laryngeal cancer is about 2.04/100 000, among which the incidence of male is higher than that of female. In the early stage of the disease, patients will have clinical manifestations of hoarseness. At the same time, it is difficult to be found in clinical practice because blood and lymphatic metastasis are rare in the early stage [1]. Laryngeal cancer is associated with a variety of factors, including age, smoking, alcohol consumption, environmental pollution, family history, and glutathione S-transferase M1 gene deletion. Therefore, for the prevention and treatment of early glottic laryngeal cancer, it is particularly important to ensure that you do not smoke, drink, eat hot and spicy food, and have regular physical examination [2, 3]. The early glottic carcinoma in clinic mainly invades the glottic tissue of the larynx. Clinically, glottic laryngeal carcinoma can be divided into three stages: Tis stage, T1a stage, and T1b stage, and a small number of lesions are limited to T2 stage [4, 5]. Because of the large trauma area of open surgery, and some patients need to take endotracheal intubation for a long time to maintain treatment, and the body tolerance is poor, the clinical promotion of open surgery is greatly limited by the difference of patients' physical quality [6–8]. The main aim of laryngeal cancer treatment is to completely remove the tumor tissue and preserve laryngeal function as much as possible. CO_2_ laser has been applied in laryngeal microsurgery for glottic laryngeal carcinoma since 1970s. Plasma radiofrequency ablation is a new minimally invasive surgical method. These two surgical methods have been applied in microsurgery of otorhinolaryngology [9]. It is difficult to ensure the safety edge because to its wide knife head and limited operation in the throat; thus, it cannot cut as accurately as a CO_2_ laser. Despite the fact that several studies have validated the usefulness of the two minimally invasive procedures, there is still debate about their efficacy [10]. The significance of this meta-analysis is to obtain the analysis results by comparing various outcome indicators of the two surgical methods through large-scale evidence-based medical data, to provide evidence-based medical evidence for clinicians to choose appropriate surgical methods according to the characteristics of patients with early glottic laryngeal carcinoma.

The article "Meta-Analysis of Low Temperature Plasma Radiofrequency Ablation and CO2 Laser Surgery on Early Glottic Laryngeal Carcinoma" was published in 2022. Journal: Comput Math Methods Med.

The main body of this study is as follows:

Section 1-Data and Methods: this section first introduces the literature retrieval methods used in this study; then, based on the purpose of the study, the inclusion and exclusion criteria of the literature are set, and the quality of the literature is evaluated; finally, the relevant data are extracted, and the statistical methods used in this study are described

Section 2–Results is as follows: this section evaluates the quality of the included literature based on the screening results of the literature and finally obtains the results of the meta-analysis

Section 3-Discussion: based on the results of the meta-analysis in Section 2, this section discusses the relevant issues

Section 4-Conclusion: final conclusion of this study

## 2. Data and Methods

### 2.1. Retrieval Methods

Two evaluators search for published domestic and foreign controlled trials. There is a computer retrieval of PubMed, Embase, Medline, VIP, Wanfang, and CNKI databases. The retrieval period is from database construction to August 31, 2021. If the outcome data report is not available or the original data is missing, send a note to the author requesting the data and including as much of the needed literature as feasible.

### 2.2. Literature Inclusion and Exclusion Criteria

In accordance with PRISMA (Preferred Reporting Items for Systematic Reviews and Meta-Analyses) principle, 2 evaluators independently screen, include, and exclude literatures for multiple times by reading the key words, abstract, and full text of literatures in detail.

Inclusion criteria were as follows: ① the patients are confirmed to have primary early laryngeal carcinoma or precancerous lesion by pathologic and cytological examination, and none of them undergo surgery or radiotherapy, ② clinical and radiographic examinations reveal no distant metastases or lymph node metastasis, and ③ the types of studies include randomized controlled trials and retrospective studies.

Exclusion criteria were as follows: ① raw data reports are incomplete, and authors cannot be contacted, ② duplicate studies with incomplete data, or multiple studies from the same center with duplicate data, the most recent study will prevail, and ③ investigate the efficacy of single treatment such as low-temperature plasma radiofrequency ablation of glottic carcinoma under supported laryngoscope or CO_2_ laser glottic carcinoma resection.

### 2.3. Literature Quality Evaluation

The included literatures are evaluated by two reviewers according to the Cochrane risk assessment criteria for bias (2016 edition. It is one of the most common bias risk assessment tools in the field of evidence-based medicine. It is mainly applicable to randomized controlled trials (RCTs)). The evaluation includes the following: ① whether a randomized controlled study, ② whether there is a distribution plan, ③ whether to perform blinding, ④ integrity of resulting data, and ⑤ other bias [11].

The article "Meta-Analysis of Low Temperature Plasma Radiofrequency Ablation and CO2 Laser Surgery on Early Glottic Laryngeal Carcinoma" was published in 2022. Journal: Comput Math Methods Med.

### 2.4. Data Extraction

Two evaluators independently screen the literature in the search results to determine potential relevance. If both parties fail to form a unified understanding, a third party can be invited to participate in the discussion to help make a decision. Literature screening is as follows: first, read the title and abstract of the literature for preliminary screening. Then, follow the established inclusion criteria and exclusion criteria to screen the literature and finally obtain the literature that meets the research objectives.

### 2.5. Statistical Method

Meta-analysis is performed using Review Manager5.3 software provided by the Cochrane collaboration for data synthesis, and the test level is *α* = 0.05. OR (odds ratio) is used for combined analysis for counting data. If the measurement tools are the same, MD (weighted mean difference) is used for continuous data analysis. SMD (standard mean difference) is used for analysis if the measurement tools are different, and 95% confidence intervals (CI) are calculated for all analyses. *χ*^2^ test is used to analyze heterogeneity. In *Q* test and *I*^2^ test, *P* > 0.1 and *I*^2^ < 50% are regarded as homogeneity, and fixed effect model is used to analyze heterogeneity [12]. *P* < 0.05 is considered statistically significant. The sensitivity analysis method is one by one elimination.

## 3. Results

This section evaluates the quality of the included literature based on the screening results of the literature and finally obtains the results of the meta-analysis.

### 3.1. Results of Literature Screening and the Basic Information of Included Studies

A total of 47 relevant literatures were retrieved using the above retrieval methods, comprising 35 Chinese literatures and 12 international literatures. After reading the full texts, 9 articles were included according to the criteria.

Gender and age differences between the observation and control groups are not statistically significant (*P* > 0.05). Outcome indicators included the following: ① recurrence rate, ② intraoperative blood loss, ③ operation time, ④ postoperative pain degree, and ⑤ postoperative mucosal recovery. Basic information of included literature is shown in Table 1.

### 3.2. Methodological Quality Evaluation of Included Studies

The included literature includes 6 RCTS and 3 RCS. Among the 9 RCTS, 1 is double-blind, and 1 is single-blind. The truncated data of 1 of all the studies are incomplete, but the reasons could be explained. The quality of the included literature meets the requirements of this study in conclusion. Bias risk analysis is shown in Figure 1.

The article "Meta-Analysis of Low Temperature Plasma Radiofrequency Ablation and CO2 Laser Surgery on Early Glottic Laryngeal Carcinoma" was published in 2022. Journal: Comput Math Methods Med.

The total score of 3 RCS scores was ≥7 points, see Table 2 for the quality evaluation of RCS documents.

### 3.3. Results of Meta-Analysis

Combined with the clinical indicators concerned about the treatment of early glottic laryngeal cancer, this study obtained the research results on the following seven indicators (Figure 2): ① recurrence rate, ② intraoperative blood loss, ③ postoperative pain degree, ④ operation time, ⑤ postoperative mucosal recovery, ⑥ sensitivity analysis, and ⑦ publication bias analysis.

### 3.4. Recurrence Rate

Recurrence rates are reported in seven literatures. In interstudy heterogeneity test: *P* = 0.624, *I*^2^ = 0%, fixed effect model analysis shows that there is no significant difference in recurrence rate between low temperature plasma radiofrequency ablation and CO_2_ laser ablation (OR = 0.80, 95% CI (0.35, 1.29), *P* = 0.371). Results of meta-analysis on recurrence rate are shown in Table 3.

### 3.5. Blood Loss in Intraoperative

Intraoperative blood loss is reported in 5 literatures, and heterogeneity test of each study is as follows: *P* = 0.03, *I*^2^ = 67%. Low temperature plasma radiofrequency ablation results in more intraoperative blood loss than CO_2_ laser ablation (SMD = −0.71, 95% CI (0.08, 0.82), *P* = 0.01). Meta-analysis results of intraoperative blood loss are shown in Table 4.

### 3.6. Postoperative Pain Degree

There are five reports on postoperative pain in two treatments: *P* = 0.04, *I*^2^ = 64%. Between low temperature plasma radiofrequency ablation and CO_2_ laser ablation (SMD = −0.21, 95% CI (-0.44, 0.10), *P* = 0.134) has no significant difference in postoperative pain (Table 5).

### 3.7. Operation Time

Operative time is reported in nine articles: *P* < 0.01, *I*^2^ = 95%. The operative time of low temperature plasma radiofrequency ablation is significantly shorter than CO_2_ laser ablation (SMD = −2.38, 95% CI (-3.91, -1.62), *P* < 0.01) (Table 6).

### 3.8. Postoperative Mucosal Recovery

There are two reports on postoperative mucosal recovery: *P* = 0.328, *I*^2^ = 2%. Low temperature plasma radiofrequency ablation was significantly better than CO_2_ laser ablation in postoperative mucosal recovery (OR = 5.49, 95% CI (2.36, 10.18), *P* < 0.01), see Table 7 for the above analysis results:

### 3.9. Sensitivity Analysis

In meta-analysis of operative time and postoperative vocal quality, there is no significant difference in the combined results before and after elimination. *I*^2^ is still greater than 50% (*I*^2^ = 69%) when the study of Shuang et al. is excluded, but the combined results of META analysis showed significant differences (SMD = 0.38, 95% CI (0.17, 0.28), *P* = 0.01). In the meta-analysis of postoperative pain, *I*^2^ decreases to 17% after removing the study of Yuke et al., and the combined results of meta-analysis still show no difference.

The article "Meta-Analysis of Low Temperature Plasma Radiofrequency Ablation and CO2 Laser Surgery on Early Glottic Laryngeal Carcinoma" was published in 2022. Journal: Comput Math Methods Med.

### 3.10. Publication Bias Analysis

Figure 3 shows a funnel plot of the operative time and recurrence rate for cryogenic plasma radiofrequency ablation and CO_2_ laser excision for early glottic laryngeal cancer and Figure 4.

## 4. Discussion

Patients with early glottic laryngeal cancer have no obvious clinical signs and are accompanied by adverse symptoms. Early treatment is often ignored. For early glottic laryngeal carcinoma, if timely diagnosis and surgical intervention, the prognosis is better [22]. Open surgery, on the other hand, has a big wound area, poor tolerance, slow postoperative recovery, and a wide range of resection, and postoperative breathing, swallowing, and vocalization functions are frequently impacted to variable degrees, lowering quality of life [23]. Therefore, it is difficult to popularize the pioneering operation in the treatment of patients with early glottic laryngeal cancer [24]. CO_2_ laser is a kind of gas molecular laser that can be continuously emitted by invisible light and far infrared spectrum. The tissue is vaporized instantly after contacting the high energy laser beam. It has the advantages of accurate target and rapid treatment [25, 26]. However, the linear beam of CO_2_ laser may increase the risk of postoperative recurrence due to the obscuring of visual field caused by poor exposure during surgery. Compared with CO_2_ laser, plasma is a new surgical method for early glottic laryngeal carcinoma with a shorter time. In addition, the plasma cutter head used in plasma radiofrequency ablation has the functions of ablation, cutting, and hemostasis. The operation is convenient, and the plasma knife head can be bent to a narrow space and cut off the lesion that is difficult to be handled by ordinary surgery [27, 28]. The basic frequency perturbation, amplitude perturbation, and harmonic noise ratio are used in a meta-analysis of postoperative vocal quality indicators to reflect the postoperative voice quality of patients. The fundamental frequency perturbation reflects the roughness of the sound, the amplitude perturbation reflects the hoarseness of the sound, and the harmonic noise ratio is related to the sound quality [29].

## 5. Conclusion

In conclusion, low temperature plasma radiofrequency ablation is superior to CO_2_ laser surgery in the treatment of early glottic laryngeal carcinoma in terms of operative time and postoperative mucosal recovery. In terms of postoperative pain, plasma radiofrequency ablation was less painful than C0_2_ laser, and the subjective and objective voice function recovered better. However, low temperature plasma radiofrequency ablation has more intraoperative blood loss, and there is no significant difference in recurrence rate and postoperative pain degree between the two treatments. In a comprehensive comparison, low-temperature plasma radiofrequency ablation for early glottic laryngeal cancer has the advantages of convenient operation, hemostasis, fast wound healing, and little damage to the surrounding tissues, which has the value of clinical promotion.

The article "Meta-Analysis of Low Temperature Plasma Radiofrequency Ablation and CO2 Laser Surgery on Early Glottic Laryngeal Carcinoma" was published in 2022. Journal: Comput Math Methods Med.

## Figures and Tables

**Figure 1:** Bias risk analysis.

**Figure 2:** Results of meta-analysis.

**Figure 3:** Funnel plot of operation time.

**Figure 4:** Funnel plot of recurrence rate.

**Table 1:** Basic information of included literature.

Included in the study	Published year	Interventions	Sample size	Gender (male/female)	Age	Observation target
Semmler et al. [13]	2011	Radio frequency group	93	79/14	60.33 ± 1.25	①, ③, ④
		Laser group	93	77/16	62.19 ± 10.13	
Liu Jianyong et al. [14]	2014	Radio frequency group	42	35/7	63.33 ± 10.88	①, ②, ③, ④
		Laser group	42	32/10	65.40 ± 10.14	
Shuang et al.[15]	2015	Radio frequency group	37	26/11	56.79 ± 9.91	②, ③
		Laser group	37	27/10	57.15 ± 10.52	
Mourad et al. [16]	2016	Radio frequency group	30	21/9	51.44 ± 8.76	②, ③, ⑤
		Laser group	30	23/7	54.23 ± 7.21	
Jun et al. [17]	2017	Radio frequency group	47	39/8	58.15 ± 8.41	①, ③, ④
		Laser group	46	36/10	57.29 ± 9.08	
Jinhui and Chengyu [18]	2018	Radio frequency group	64	51/13	55.26 ± 2.45	①, ②, ③, ④
		Laser group	64	50/14	56.79 ± 4.51	
Yuke et al. [19]	2019	Radio frequency group	52	40/12	61.19 ± 6.54	①, ③, ④
		Laser group	52	38/14	62.37 ± 6.76	
Yong et al. [20]	2020	Radio frequency group	48	37/11	60.04 ± 6.99	①, ②, ③
		Laser group	47	40/7	59.63 ± 4.58	
Bin et al. [21]	2021	Radio frequency group	33	24/9	58.33 ± 9.36	①, ③, ⑤
		Laser group	33	23/10	59.17 ± 8.64	

**Table 2:** Quality evaluation of RCS included literature.

Included in the study	Grouping method	Report lost to follow-up	Blind method	Diagnostic criteria	Baseline	Confounding factor control	Total score
Liu Jianyong et al.	No specific description	No lost to follow-up	Not mentioned	The “gold standard” diagnosis	Well described, well balanced	Appropriate	9
Jun et al.	No specific description	No lost to follow-up	Not mentioned	The “gold standard” diagnosis	Well described, well balanced	Appropriate	9
Yuke et al.	No specific description	Reported lost to follow-up and the rate of lost to follow-up <10%	Not mentioned	Not described	Well described, well balanced	Appropriate	8

The article "Meta-Analysis of Low Temperature Plasma Radiofrequency Ablation and CO2 Laser Surgery on Early Glottic Laryngeal Carcinoma" was published in 2022. Journal: Comput Math Methods Med.

**Table 3:** Results of meta-analysis on recurrence rate.

Study or subgroup	Radio frequency group		Laser group		Weight	Odds ratio, *M*-*H*, fixed, 95% CI
	Events	Total	Events	Total		
Semmler et al.	12	93	11	93	36.24%	0.74 [0.21, 2.06]
Liu Jianyong et al.	1	42	3	42	9.21%	0.13 [0.03, 2.87]
Jun et al.	2	47	1	46	1.67%	4.98 [0.23, 1113.13]
Jinhui and Chengyu	7	64	5	64	17.35%	1.784 [0.36, 4.56]
Yuke et al.	2	52	5	52	5.29%	0.36 [0.08, 2.08]
Yong et al.	2	48	3	47	5.12%	0.53 [0.08, 6.14]
Bin et al.	1	33	0	33	25.12%	0.754 [0.42, 1.89]
Total (95% CI)		379		377	100.00%	0.80 [0.35, 1.29]
Total events	27		28			

Heterogeneity: chi^2^ = 4.82, df = 7 (*P* = 0.624); *I*^2^ = 0%. Test for overall effect: *Z* = 0.88 (*P* = 0.371).

**Table 4:** Meta-analysis results of intraoperative blood loss.

Study or subgroup	Radio frequency group		Laser group		Weight	Odds ratio, *M*-*H*, fixed, 95% CI
	Mean ± SD	Total	Mean ± SD	Total		
Liu Jianyong et al.	10.28 ± 2.62	42	10.67 ± 2.34	42	22.17%	-0.98 [-0.34, 0.31]
Shuang et al.	11.33 ± 2.45	37	10.42 ± 6.87	37	18.09%	0.24 [-0.23, 0.65]
Mourad et al.	10.27 ± 2.37	30	8.52 ± 2.17	30	23.11%	0.87 [0.24, 1.35]
Jinhui and Chengyu	10.30 ± 2.39	64	8.97 ± 2.36	64	17.09%	0.64 [0.92, 1.22]
Yong et al.	10.32 ± 0.79	48	9.37 ± 0.45	47	19.54%	0.67 [0.28, 1.35]
Total (95% CI)		221		220	100.00%	0.43 [0.08, 0.82]

Heterogeneity: tau^2^ = 0.09; Chi^2^ = 11.37, df = 5 (*P* = 0.03); *I*^2^ = 67%. Test for overall effect: *Z* = 2.49 (*P* = 0.01).

**Table 5:** Results of meta-analysis of postoperative pain degree.

Study or subgroup	Radio frequency group		Laser group		Weight	Odds ratio, *M*-*H*, fixed, 95% CI
	Mean ± SD	Total	Mean ± SD	Total		
Semmler et al.	2.78 ± 0.37	93	2.88 ± 0.98	93	19.89%	-0.07 [-0.35, 0.26]
Liu Jianyong et al.	2.76 ± 1.08	42	2.90 ± 0.25	42	17.98%	-0.31 [-0.65, 0.09]
Jun et al.	2.67 ± 0.98	47	3.09 ± 1.12	46	13.12%	-0.32 [-0.76, 0.29]
Jinhui and Chengyu	2.86 ± 0.14	64	2.77 ± 0.55	64	15.09%	0.16 [-0.45, 0.65]
Yuke et al.	2.84 ± 0.63	52	3.18 ± 0.47	52	33.92%	-0.75 [-1.25, -3.08]
Total (95% CI)		298		297	100.00%	0.16 [-0.44, 0.10]

Heterogeneity: tau^2^ = 0.07; chi^2^ = 13.25, df = 5 (*P* = 0.04); *I*^2^ = 64%. Test for overall effect: *Z* = 1.38 (*P* = 0.134).

**Table 6:** Results of meta-analysis of operation time.

Study or subgroup	Radio frequency group		Laser group		Weight	Odds ratio, *M*-*H*, fixed, 95% CI
	Mean ± SD	Total	Mean ± SD	Total		
Semmler et al.	1.25 ± 0.44	93	1.08 ± 0.29	93	11.23%	-2.09 [-2.33, -1.79]
Liu Jianyong et al.	2.69 ± 0.15	42	1.82 ± 0.39	42	10.32%	-2.87 [-2.98, -1.09]
Shuang et al.	1.04 ± 0.16	37	1.23 ± 0.17	37	3.89%	-3.44 [-4.09, -2.41]
Mourad et al.	1.09 ± 0.39	30	1.46 ± 0.18	30	10.08%	22.87 [16.43, 0.81]
Jun et al.	2.63 ± 0.34	47	3.94 ± 0.58	46	10.67%	-1.82 [-0.24, -1.79]
Jinhui and Chengyu	5.61 ± 0.28	64	4.76 ± 0.33	64	10.59%	-1.23 [-0.24, -1.79]
Yuke et al.	2.65 ± 0.18	52	3.58 ± 0.54	52	10.49%	-1.82 [-2.44, -1.79]
Yong et al.	4.81 ± 0.18	48	5.76 ± 0.34	47	11.34%	-1.86 [-1.53, -3.10]
Bin et al.	21.32 ± 3.05	33	22.14 ± 3.78	33	21.39%	-4.76 [-5.09, -4.01]
Total (95% CI)		446		444	100.00%	-2.06 [-3.91, -1.62]

Heterogeneity: tau^2^ = 2.78; chi^2^ = 225.98, df = 9 (*P* < 0.01); *I*^2^ = 95%. Test for overall effect: *Z* = 5.72 (*P* ≤ 0.01).

The article "Meta-Analysis of Low Temperature Plasma Radiofrequency Ablation and CO2 Laser Surgery on Early Glottic Laryngeal Carcinoma" was published in 2022. Journal: Comput Math Methods Med.

**Table 7:** Results of meta-analysis of postoperative mucosal recovery.

Study or subgroup	Radio frequency group		Laser group		Weight	Odds ratio, *M*-*H*, fixed, 95% CI
	Events	Total	Events	Total		
Mourad et al.	24	30	16	30	74.38%	4.35 [2.09, 9.02]
Bin et al.	27	33	19	33	25.62%	25.18 [2.31, 23.09]
Total (95% CI)		63		63	100.00%	5.49 [2.36, 10.18]
Total events	51		35			

Heterogeneity: chi^2^ = 2.09, df = 2 (*P* = 0.328); *I*^2^ = 2%. Test for overall effect: *Z* = 5.19 (*P* < 0.01).

## Data Availability

The data used to support the findings of this study are included within the article.

## References

[1] Testa D., Guerra G., Conzo G. (2013). Glottic-subglottic adenoid cystic carcinoma. A case report and review of the literature[J]. *BMC Surgery*.

[2] Chunhong Z., Yujie L., Min Y. (2015). Comparison of CO2 laser and plasma radiofrequency ablation in the treatment of early glottic laryngeal carcinoma. *Journal of Audiology and Speech Disorders*.

[3] Hua X., Haiping Z., Le L. (2016). Comparison between radiofrequency ablation combined with chemotherapy and surgery combined with chemotherapy in the treatment of glottic laryngeal carcinoma[J]. *China Medical Guide*.

[4] Yong W., Jianfeng L. (2021). To explore the clinical effect of carbon dioxide laser therapy on early glottic laryngeal cancer [J]. *Chinese Medical Abstracts (otorhinolaryngology)*.

[5] Xiaoling J. (2022). Effect of plasma ablation assisted by supporting laryngoscope and endoscope on postoperative rehabilitation and voice function of patients with early glottic laryngeal cancer [J]. *Medical theory and practice*.

[6] Peng G., Xiongwei L. (2018). Effect of low temperature plasma radiofrequency ablation on early glottic laryngeal carcinoma [J]. *Journal of Practical Cancer*.

[7] Fei D., Yi C., Yanchen C., Huiwen Z. (2021). Clinical effect of carbon dioxide laser treatment of early glottic laryngeal carcinoma under support laryngoscope [J]. *Chinese contemporary medicine*.

[8] Meijuan L. V., Yixing L., Gendong Y. (2022). Treatment of glottic laryngeal carcinoma by low temperature plasma radiofrequency ablation under microsupport laryngoscope [J]. *Zhejiang trauma surgery*.

The article "Meta-Analysis of Low Temperature Plasma Radiofrequency Ablation and CO2 Laser Surgery on Early Glottic Laryngeal Carcinoma" was published in 2022. Journal: Comput Math Methods Med.

[9] Nguyen-Tan P. F., Le Q. T., Quivey J. M. (2001). Treatment results and prognostic factors of advanced T3--4 laryngeal carcinoma: the University of California, San Francisco (UCSF) and Stanford University Hospital (SUH) experience[J]. *International Journal of Radiation Oncology • Biology • Physics*.

[10] Quansheng L., Yiyang H., Wang L., Jiang W., Hongwei L. (2020). Effect of transoral CO_2 laser, partial laryngectomy and low temperature plasma radiofrequency ablation on glottic laryngeal carcinoma [J]. *Chinese Oncology Clinic and Rehabilitation*.

[11] Huiling T., Jialiang G. (2021). Research progress in minimally invasive treatment of early glottic laryngeal carcinoma[J]. *Cancer Progress*.

[12] Juntao H., Lixin C., Linrong W., Ting Y., Yi S. (2021). Meta-analysis of the efficacy of cryogenic plasma radiofrequency ablation and carbon dioxide laser in the treatment of early glottic laryngeal carcinoma [J]. *Chinese Journal of Cancer Prevention and Treatment*.

[13] Semmler M., Keck T., Reiter R., Gruen P. M. (2011). Endolaryngeal posterior mucosal flap for surgical repair of posterior glottic stenosis. *Auris Nasus Larynx*.

[14] Jianyong L., Jianbin L., Menglin L., Yue X., Qi Y., Yifang Y. (2014). Clinical effect of low temperature plasma radiofrequency ablation on early glottic laryngeal carcinoma[J]. *Chinese Journal of Integrated Traditional and Western Medicine Otolaryngology*.

[15] Yu S., Chao L., Yongwang H., Shuang W. (2015). Comparison of cryogenic plasma radiofrequency ablation and CO2 laser in the treatment of early glottic laryngeal carcinoma[J]. *Journal of Audiology and Speech Disorders*.

[16] Mourad M., Dezube A., Moshier E., Shin E. (2016). Geographic trends in management of early-stage laryngeal cancer. *Laryngoscope*.

[17] Jun D., De H., Zhibin C. (2017). Clinical observation of CO2 laser combined with cryogenic plasma radiofrequency ablation in the treatment of early glottic laryngeal carcinoma with preinvolvement[J]. *Chinese Oncology Clinic and Rehabilitation*.

[18] Jinhui Z., Chengyu W. (2018). Effects of CO2 laser and plasma radiofrequency ablation on surgical indicators, pain and recurrence of early glottic laryngeal carcinoma [J]. *Chinese General Practice*.

[19] Yuke D., Yujie L., Wei H. (2019). Effects of CO2 laser combined with plasma radiofrequency ablation on cytokine levels in early glottic laryngeal carcinoma[J]. *Chinese Journal of Modern Medicine*.

[20] Yong T., Yuzi J., Jiqing M. (2020). The prognostic value of low temperature plasma radiofrequency ablation,CO2 laser and laryngeal dehiscence in the treatment of early glottic laryngeal carcinoma in the elderly by serum thymidine kinase 1[J]. *Journal of Practical Cancer*.

The article "Meta-Analysis of Low Temperature Plasma Radiofrequency Ablation and CO2 Laser Surgery on Early Glottic Laryngeal Carcinoma" was published in 2022. Journal: Comput Math Methods Med.

[21] Bin H., Weiping H., Zhongpu Y., Yonggang L. (2021). Effect and influencing factors of low temperature plasma radiofrequency ablation in the treatment of early glottic laryngeal carcinoma [J]. *Cancer Progress*.

[22] Furusaka T., Susaki Y., Saito T., Katsura Y., Ikeda M. (2013). Long-term follow-up and salvage surgery in patients with T2N0M0 squamous cell carcinoma of the glottic larynx following concurrent chemoradiation therapy with cisplatin and 5-fluorouracil for laryngeal preservation. *Acta Oto-Laryngologica*.

[23] Jianli C., Zhiqiang Z. (2019). Effects of cryogenic plasma radiofrequency ablation on VAS score and complications of early glottic laryngeal carcinoma [J]. *Modern Digestion & Intervention*.

[24] Min Z., Yujun L. (2021). Research progress in the treatment of early glottic laryngeal carcinoma [J]. *Journal of practical cardio cerebrovascular diseases*.

[25] Jiaming Y., Xufen Y., Yali Z. (2022). Discussion on CO under microsupport laryngoscope_ clinical effect of laser therapy on early glottic laryngeal carcinoma [J]. *Yunnan medicine*.

[26] Ming L. (2018). CO2 laser therapy for suprglottic laryngeal carcinoma [J]. *Journal of Otolaryngology, Shandong University*.

[27] Dasong L., Yongjun F., Chunrong Z., Mingjing W. (2016). Comparative analysis of the efficacy of endoscopic low temperature plasma radiofrequency ablation and conventional laryngeal dehysis in the treatment of early glottic laryngeal carcinoma[J]. *Journal of Clinical Pathology*.

[28] Weixing L., Gui C., Lijuan S., Wenjing L., Xiaowen Z. (2022). Plasma radiofrequency ablation and Co_ effect of laser surgery on pain and recurrence in patients with early glottic laryngeal cancer [J]. *Chinese Journal of modern medicine*.

[29] Weixing L., Gui C., Lijuan S. (2020). Metaanalysis of cryogenic plasma radiofrequency ablation and CO 2 laser therapy for early glottic laryngeal carcinoma [J]. *Chinese Journal of Biomedical Engineering*.

